The article "Relationship between Severity of Disease and Postoperative Neurological Recovery in Patients with Cervical Spondylotic Myelopathy Combined with Developmental Spinal Stenosis" was retracted in 2023. Reasons: signs of a paper mill; suspected computer-generated content; unreliable results or conclusions; concerns about the data.

# Relationship between Severity of Disease and Postoperative Neurological Recovery in Patients with Cervical Spondylotic Myelopathy Combined with Developmental Spinal Stenosis

**DOI:** 10.1155/2022/9800993

**Published:** 2022-09-27

**Authors:** Shuai Wang, Jingtao Zhang, Shuo Peng, Junming Cao, Wei Du, Yu Zhang, Zhixin Gong, Li Zhang, Yong Shen

**Affiliations:** ^1^Department of Orthopaedics, The Third Hospital of Hebei Medical University, Shijiazhuang, China; ^2^Scientific Research Division, The Third Hospital of Hebei Medical University, Shijiazhuang, China; ^3^Department of Orthopaedics, Hebei Geriatric Hospital, Qinhuangda, China; ^4^Department of Spine surgery, The Third Hospital of Hebei Medical University, Shijiazhuang, China

## Abstract

**Objective:**

The study aimed to investigate the correlation between the severity of disease and postoperative neurological recovery in patients with cervical spondylotic myelopathy (CSM) combined with developmental spinal stenosis.

**Methods:**

A retrospective analysis of the clinical data of 114 CSM patients combined with developmental spinal stenosis admitted to our hospital from June 2019 to June 2020 was performed. All of the patients who underwent posterior cervical unidoor vertebroplasty were divided into the mild, moderate, and severe groups according to the Torg–Pavlov ratio. The clinical data including patients' age, course of spinal cord high signal change, and first onset age were collected. The recovery time, preoperative, and postoperative Japanese Orthopaedic Association (JOA) scores of patients in each group were compared with the calculation of the improvement rate. The correlation between the severity of disease and postoperative neurological recovery in CSM patients combined with developmental spinal stenosis was analyzed by Pearson correlation. The factors influencing postoperative neurological recovery were analyzed using multivariate logistic regression analysis. The receiver operating characteristic curve (AUC) was used to evaluate the value of each influencing factor in predicting postoperative recovery.

**Results:**

Significant differences were observed in the proportion of linear hyperintensity changes in the spinal cord, the age of first onset, the course of the disease, and the Torg–Pavlov ratio among the mild, moderate, and severe groups (*P*  <  0.05). The postoperative recovery time of the moderate and severe groups was significantly higher than that of the mild group, while the preoperative JOA score was significantly lower than that of the mild group. On the other hand, the postoperative recovery time of the severe group was prominently higher than that of the moderate group, whereas the preoperative JOA score was observably lower than that of the moderate group (*P*  <  0.05). Pearson correlation analysis showed that the postoperative recovery time was significantly negatively correlated with the Torg–Pavlov ratio, age at first onset, and disease course (*r* = −0.359, −0.502, −0.368, *P*  <  0.05), while it was positively correlated with spinal cord linear high-signal changes (*r* = 0.641, *P*  <  0.05). Multifactorial logistic regression analysis revealed that the Torg–Pavlov ratio, age at first onset, and disease course were protective factors, while spinal cord linear high-signal alterations were risk factors affecting the recovery time of postoperative neurological function (*P*  <  0.05). The area under the curve (AUC) of the Torg–Pavlov ratio, linear hyperintensity changes in the spinal cord, age at first onset, and disease duration in predicting the postoperative neurological recovery time were 0.794, 0.767, 0.772, and 0.802, respectively. The AUC predicted by the combined detection of each factor was 0.876, which was better than the area under the curve of single prediction.

The article "Relationship between Severity of Disease and Postoperative Neurological Recovery in Patients with Cervical Spondylotic Myelopathy Combined with Developmental Spinal Stenosis" was retracted in 2023. Reasons: signs of a paper mill; suspected computer-generated content; unreliable results or conclusions; concerns about the data.

**Conclusion:**

Patients with CSM combined with developmental spinal stenosis were characterized by younger age of onset, a short course of the disease, and linear changes in the spinal cord high signal. The degree of developmental spinal stenosis may affect the postoperative recovery time of neurological function in CSM patients but had little effect on postoperative neurological recovery. The Torg–Pavlov ratio, age of first onset, course of the disease, and changes in the spinal cord linear hyperintensity were the factors that affected postoperative neurological recovery, which may provide a basis for reasonably predicting a postoperative neurological recovery in patients with CSM combined with developmental spinal stenosis.

## 1. Introduction

Cervical spondylotic myelopathy (CSM) is a chronic degenerative cervical spondylosis with a high clinical incidence rate, which is induced by the degeneration of the cervical vertebrae connecting structure, leading to spinal cord compression or spinal cord ischemia and then spinal cord dysfunction. The early symptoms of CSM are not obvious; thus, most patients already have had obvious limb symptoms at the first time of hospital visit, which eventually leads to serious disablement. CSM is also one of the most common causes of adult spastic paraplegia, which greatly reduces the quality of life of patients and brings a huge economic burden to families and society [1, 2]. With the change of work style and the aggravation of population aging in recent years, the number of CSM patients has gradually increased accompanied by a younger trend, which has attracted the attention of medical practitioners all over the world [3].

The article "Relationship between Severity of Disease and Postoperative Neurological Recovery in Patients with Cervical Spondylotic Myelopathy Combined with Developmental Spinal Stenosis" was retracted in 2023. Reasons: signs of a paper mill; suspected computer-generated content; unreliable results or conclusions; concerns about the data.

Surgical treatment is a common treatment for CSM at present, among which posterior open-door laminoplasty of the cervical spine is a more mature clinical treatment. It not only relieves the compression of the spinal cord but also maintains the stability of the spine; thus, it has been accepted by patients due to its good therapeutic effect [4, 5]. However, there are some uncertainties during the recovery of postoperative neurological function, since some patients are accompanied by early neck pain, postoperative axial symptoms, and C5 nerve root paralysis. Developmental spinal stenosis is one of the important factors in the occurrence and development of CSM, which is induced by the narrow inner diameter of the cervical spinal canal during individual development. Developmental spinal stenosis can not only reduce the threshold of symptoms and signs but also lead to cervical degeneration. Moreover, CSM patients with developmental spinal stenosis have earlier clinical symptoms and signs than those without developmental spinal stenosis [6]. Relevant data show that the incidence of developmental spinal stenosis increases with the age of the patient, which can cause spinal cord compression or ischemic changes, resulting in numbness of the limbs, unsteady walking, positive pathological signs, and other symptoms of myelopathy [7]. However, there is no research report on whether the degree of developmental spinal canal stenosis affects the recovery of postoperative neurological function in patients with CSM.

In this study, 114 CSM patients with developmental spinal stenosis admitted to our hospital from June 2019 to June 2020 were selected as the objects, to analyze the correlation between the condition of CSM patients combined with developmental spinal stenosis and the recovery of postoperative neurological function.

## 2. Materials and Methods

### 2.1. General Materials

A total of 114 CSM patients with developmental spinal stenosis admitted to our hospital from June 2019 to June 2020 were selected as the objects. Inclusion criteria were as follows: (1) All patients met the diagnostic criteria for CSM in the National Symposium on Cervical Spondylosis, and cervical degenerative changes were shown in X-ray; (2) all patients underwent posterior open-door laminoplasty; (3) the patients and their family members were informed and had good compliance. They could cooperate with the examination and treatment. The patients were followed-up for more than 1 year and signed the informed consent form. Exclusion criteria were as follows: (1) patients with severe dysfunction of important organs; (2) patients combined with nervous system damage caused by other reasons or other cervical diseases. According to the Torg–Pavlov ratio, the patients were divided into the mild group (0.65 < Torg–Pavlov ratio ≤0.75), moderate group (0.55 < Torg–Pavlov ratio ≤0.65), and severe group (Torg–Pavlov ratio ≤0.55). All the experiments were approved by the ethics committee of the hospital. The process of general material selection is shown in Figure 1.

The article "Relationship between Severity of Disease and Postoperative Neurological Recovery in Patients with Cervical Spondylotic Myelopathy Combined with Developmental Spinal Stenosis" was retracted in 2023. Reasons: signs of a paper mill; suspected computer-generated content; unreliable results or conclusions; concerns about the data.

### 2.2. Methods

All patients underwent posterior open-door laminoplasty of the cervical spine. The patient was intubated under general anesthesia in the prone position. An incision from the second cervical vertebra to the seventh cervical vertebra was made after paving the sterile sheet. We separated the spinous processes and cut off the C (2–3) to C (6–7) interspinous ligaments. We polished the junction of the vertebral lamina and lateral mass, and we selected the side with heavier symptoms on the door opening side and the side with lighter symptoms on the hinge side. We removed the ligamentum flavum on the opening side, C (2–3) and C (6–7), opened the vertebral lamina, placed the laminoplasty plate on the opening side of C (3–6), and fixed it with a microtitanium plate or anchor screw to complete the opening. We performed the laminectomy and preserved the spinal ligament complex, which is horizontal to C7. After the nail plate was fixed well, debridement and hemostasis were performed, an artificial dura mater and a drainage tube were placed, sutured layer by layer, and the incision was covered with the sterile application. The drainage tube was placed for 48 h. After the operation, the cervical vertebrae were fixed with cervical brackets, and functional training was performed after removing the cervical brackets.

### 2.3. Outcome Measures

Clinical data: clinical data in each group, including age, spinal cord hyperintensity changes, course of the disease, age of first onset, gender, the most severely compressed segment, the Torg–Pavlov ratio, visual analog scale (VAS), high blood pressure, and smoking history were collected. Among them, the spinal cord hyperintensity changes were judged by MRI examination, which were divided into none, punctate, and linear by recording the presence or absence of T2 hyperintensity changes in the spinal cord and the longitudinal extent of hyperintensity changes. The Torg–Pavlov ratio used CT standard distance projection lateral films as the standard to measure the sagittal diameter of the spinal canal (the shortest distance from the posterior edge of the vertebral body to the line connecting the lamina) and the midsagittal diameter of the vertebral body (the line connecting the midpoints of the anterior and posterior borders of the vertebral body) for the calculation of the Torg–Pavlov ratio.

The article "Relationship between Severity of Disease and Postoperative Neurological Recovery in Patients with Cervical Spondylotic Myelopathy Combined with Developmental Spinal Stenosis" was retracted in 2023. Reasons: signs of a paper mill; suspected computer-generated content; unreliable results or conclusions; concerns about the data.

Perioperative indicators: we closely observed the patient's physical condition, recorded and compared the perioperative indicators such as intraoperative bleeding volume and operation time, and recorded the postoperative recovery time of patients in each group. The follow-up was conducted after the operation for one year. The preoperative and postoperative Japanese Orthopaedic Association (JOA) scores were compared. The JOA score included 5 items: upper limb motor function, lower limb motor function, upper limb sensory function, lower limb sensory function, and bladder function, with a total score of 17 points. The higher the score was, the lower the degree of spinal cord injury was. The JOA improvement rate was calculated according to the JOA score before and after treatment. The improvement rate = (postoperative JOA score-preoperative JOA score)/(17-preoperative JOA score) × 100%.

### 2.4. Statistical Analysis

The experimental data were analyzed using Spss20.0 software. Measurement data including the age, course of the disease, and age at first onset were expressed as ($\bar{x}$ ± *s*) and compared using repeated measures analysis of variance among three groups or the LSD-t test between the two groups. Enumeration data such as gender, spinal cord hyperintensity changes, and the most severely compressed segment were expressed in (%) and compared using the *χ*2 test. The correlation between the severity of CSM patients combined with developmental spinal stenosis and the recovery of postoperative neurological function was analyzed using Pearson correlation analysis. The factors influencing the recovery time of postoperative neurological function were analyzed by multivariate logistic regression. The receiver operating characteristic curve (AUC) was used to evaluate the value of each influencing factor in predicting postoperative recovery. *P*  <  0.05 was considered statistically significant.

## 3. Results

### 3.1. Comparison of Clinical Data and Perioperative Indexes in Each Group

There were significant statistical differences in the proportion of linear hyperintensity changes in the spinal cord, the age of first onset, the course of the disease, and the Torg–Pavlov ratio among the mild, moderate, and severe groups (*P*  <  0.05) (Table 1).

### 3.2. Comparison of Postoperative Recovery-Related Indexes in Each Group

The postoperative recovery time of patients in the moderate and severe groups was significantly higher than that of the mild group, while the preoperative JOA score was prominently lower than that of the mild group. Meanwhile, the postoperative recovery time of the patients in the severe group was observably higher than that of the moderate group, whereas the preoperative JOA score was markedly lower than that of the moderate group (*P*  <  0.05) (Table 2).

The article "Relationship between Severity of Disease and Postoperative Neurological Recovery in Patients with Cervical Spondylotic Myelopathy Combined with Developmental Spinal Stenosis" was retracted in 2023. Reasons: signs of a paper mill; suspected computer-generated content; unreliable results or conclusions; concerns about the data.

### 3.3. Correlation Analysis between Severity of Patients' Condition and Postoperative Neurological Recovery

Pearson correlation analysis showed that postoperative recovery time was negatively correlated with the Torg–Pavlov ratio, first onset age, and disease duration (*r* = −0.359, −0.502, −0.368, all *P*  <  0.05), while it was positively correlated with spinal cord linear high-signal changes (*r* = 0.641, *P*  <  0.05) (Table 3 and Figure 2).

### 3.4. Analysis of Factors Influencing the Recovery Time of Postoperative Neurological Function

Multivariate logistic regression analysis was performed with the time of postoperative neurological recovery as the dependent variable. The Torg–Pavlov ratio, linear hyperintensity changes in the spinal cord, age of first onset, and disease duration were performed as independent variables. The results showed that the Torg–Pavlov ratio, age of first onset, and duration of disease were protective factors, and linear high-signal changes in the spinal cord were risk factors affecting the recovery time of postoperative neurological function (*P*  <  0.05) (Table 4).

### 3.5. ROC Curve for Predicting the Recovery Time of Neurological Function in Patients with CSM

The four predictors in Table 4 are used as test variables to construct the ROC curve, respectively, or jointly. The area under the curve (AUC) was calculated and compared. The results showed that the AUC of the Torg–Pavlov ratio, linear hyperintensity changes in the spinal cord, age at first onset, and disease duration in predicting the postoperative neurological recovery time were 0.794, 0.767, 0.772, and 0.802, respectively. The AUC predicted by the combined detection of each factor was 0.876, which was better than the area under the curve of single prediction (Table 5 and Figure 3).

## 4. Discussion

CSM is currently the most common cervical spondylosis with the worst prognosis, which largely endangers human health [8]. The clinical manifestations of CSM vary according to the location and degree of spinal cord compression, representing abnormal limb function, unstable walking, and even quadriplegia. CSM has a high disability rate, which not only brings great pain to patients but also brings a certain degree of the medical economic burden to society and families [9, 10]. The primary cause of CSM is spinal canal stenosis caused by cervical degeneration. In addition, intervertebral disc herniation and osteophytes can directly compress the spinal cord, causing ischemia, hypoxia, and other symptoms. At present, there are no effective drugs and other nonsurgical treatment methods to relieve compression. The purpose of the operation is to relieve the spinal cord compression by expanding the spinal canal, but the postoperative neurological recovery of some CSM patients worsens [11, 12]. Therefore, this study aimed to compare the clinical characteristics of CSM patients with different developmental spinal stenosis and to further clarify the impact of developmental spinal stenosis on the specific recovery process after operation.

The article "Relationship between Severity of Disease and Postoperative Neurological Recovery in Patients with Cervical Spondylotic Myelopathy Combined with Developmental Spinal Stenosis" was retracted in 2023. Reasons: signs of a paper mill; suspected computer-generated content; unreliable results or conclusions; concerns about the data.

Developmental spinal stenosis is stenosis caused by developmental factors of the spinal canal such as short pedicles and facet joint cohesion. It does not necessarily show clinical symptoms and signs, but when the volume of the spinal canal is gradually incompatible with the spinal cord tissue, clinical symptoms may appear if secondary factors are encountered. Developmental spinal stenosis is more common in East Asian populations [13], which is one of the important factors in the pathogenesis of CSM [14]. It has been shown that the probability of developing CSM in patients with developmental spinal stenosis is significantly higher than that in the normal population. The research by Erdi et al. [15] demonstrated that spinal cord compression by intervertebral disc degeneration is a secondary factor, while developmental spinal stenosis is a pre-existing factor among the pathogenic factors of CSM. In the current study, significant statistical differences were observed in the proportion of linear hyperintensity changes in the spinal cord, the age of first onset, the course of the disease, and the Torg–Pavlov ratio among the mild, moderate, and severe groups, which indicated that patients with CSM combined with developmental spinal stenosis are characterized by younger age of onset, short course of the disease, and linear changes in the spinal cord high signal, in line with the results of the study by Özer et al. [16]. It is believed that compared with ordinary CSM patients, CSM patients with developmental spinal stenosis may be more severely ill. The reason may be related to the fact that patients with developmental spinal stenosis have less spinal canal space and are more likely to receive mechanical compression, instability, and blood flow disorders. Therefore, the onset and development of the disease are faster than those without developmental spinal stenosis.

Posterior single-door laminoplasty of the cervical spine is a common surgical treatment in clinics at present. It relieves the compression of the spinal cord and restores the stability of the spinal cord by expanding the spinal canal, pushing the spinal cord to move backward, and reducing the multilevel pressure of the spinal cord, so as to effectively restore the spinal cord function. This procedure is applicable to mild and severe multilevel intervertebral disc herniation [14, 17]. However, there is no relevant research report on the difference in postoperative neurological recovery in patients with developmental spinal stenosis. In the present study, significant differences existed in the postoperative recovery time and preoperative JOA score among the mild, moderate, and severe groups, while no significant difference was discovered in the postoperative JOA score and improvement rate, suggesting that developmental spinal stenosis may affect the recovery time of postoperative neurological function in patients with CSM, but it has less impact on the recovery of postoperative neurological function. The Pearson correlation analysis was conducted to further explore the relationship between the severity of developmental spinal stenosis and the postoperative neurological recovery of CSM patients. The results showed that the Torg–Pavlov ratio, initial age, course of the disease, and linear high-signal changes in the spinal cord were closely correlated with the postoperative recovery time, affecting the postoperative neurological recovery time of patients but had no significant correlation with the postoperative JOA score and the improvement rate. It further indicated that the postoperative recovery of CSM patients combined with developmental spinal stenosis might be slower, but no significant differences existed in the final neurological recovery of patients with different degrees of developmental spinal stenosis. The results of logistic regression analysis in this study showed that the Torg–Pavlov ratio, age at first onset, and disease duration were protective factors, while spinal cord linear hyperintensity was a risk factor affecting postoperative neurological function recovery. The ROC curve results revealed that the combination of each index had a certain predictive value for the postoperative recovery time. Relevant data show [18] that patients with severe developmental spinal stenosis progress faster and are prone to MRI spinal cord T2 high signal changes in a short time after symptoms appear. Therefore, this study suggests that such patients should be closely reviewed, the progression of the disease should be observed, and timely surgery should be performed after symptoms appear to avoid further development of the disease leading to irreversible nerve damage.

The article "Relationship between Severity of Disease and Postoperative Neurological Recovery in Patients with Cervical Spondylotic Myelopathy Combined with Developmental Spinal Stenosis" was retracted in 2023. Reasons: signs of a paper mill; suspected computer-generated content; unreliable results or conclusions; concerns about the data.

In conclusion, patients with CSM combined with developmental spinal stenosis are characterized by younger age of onset, short course of the disease, and linear changes in the spinal cord high signal. The degree of developmental spinal stenosis can affect the postoperative recovery time of neurological function in CSM patients but has little effect on postoperative neurological recovery. The Torg–Pavlov ratio, age of first onset, course of the disease, and changes in spinal cord linear hyperintensity are all factors that affect postoperative neurological recovery, which can provide a basis for reasonably predicting a postoperative neurological recovery in patients with CSM combined with developmental spinal stenosis. However, due to the short research time and the small number of samples in this experiment, the experimental results may be accidental. In the future, the experimental objects and research time will be expanded for in-depth research.

## Figures and Tables

**Figure 1:** Process of general material selection.

**Figure 2:** Pearson correlation analysis. Figure A1∼4: correlation between the postoperative JOA score and neurological recovery; Figure B1∼4: correlation between the JOA score improvement rate and neurological recovery; Figure C1∼4: correlation between the postoperative recovery time and neurological recovery.

**Figure 3:** ROC curve analysis.

**Table 1:** Comparison of clinical data and perioperative indexes in each group ($\bar{x}$ ± *s*).

Indexes		Mild group (*n* = 54)	Moderate group (*n* = 42)	Severe group (*n* = 18)	*F*	*P*
Age (year)		58.26 ± 8.15	57.89 ± 6.38	58.34 ± 10.46	0.030	0.968
Gender (cases)	Male	34 (62.96%)	23 (54.76%)	14 (77.78%)	2.861	0.239
	Female	20 (37.04%)	19 (45.24%)	4 (22.22%)		
High signal	None	22 (40.74%)	19 (45.24%)^a^	3 (16.67%)^ab^		
Changes of	Punctate change	28 (51.85%)	12 (28.57%)^a^	2 (11.11%)^ab^	21.593	<0.001
Spinal cord	Linear change	4 (7.41%)	11 (26.19%)^a^	13 (72.22%)^ab^		
Course of disease (year)		7.46 ± 1.25	5.39 ± 1.04^a^	2.15 ± 0.85^ab^	157.330	<0.001
Most severely compressed segments	C3–5 C5–7	24 (44.44%) 30 (55.56%)	22 (52.38%) 20 (47.62%)	10 (55.56%) 8 (44.44%)	0.949	0.622
First age of onset (year)		54.16 ± 5.26	56.86 ± 6.35^a^	47.15 ± 5.48^ab^	18.180	<0.001
Preoperative VAS score		1.49 ± 1.58	1.54 ± 1.26	1.46 ± 1.32	0.020	0.976
Smoking history		18 (33.33%)	15 (35.71%)	7 (38.89%)	0.194	0.907
Hypertension		16 (29.63%)	17 (40.48%)	5 (27.78%)	1.548	0.461
Torg–Pavlov ratio		0.71 ± 0.26	0.60 ± 0.28^a^	0.41 ± 0.16^ab^	9.570	<0.001
Intraoperative bleeding volume (ml)		343.19 ± 10.52	339.15 ± 15.69	335.85 ± 20.41	2.060	0.132
Time of operation (min)		172.63 ± 25.64	176.15 ± 24.15	180.15 ± 20.63	0.700	0.497

*Note*. ^a^*P*  <  0.05 compared with the mild group; ^b^*P*  <  0.05 compared with the moderate group.

The article "Relationship between Severity of Disease and Postoperative Neurological Recovery in Patients with Cervical Spondylotic Myelopathy Combined with Developmental Spinal Stenosis" was retracted in 2023. Reasons: signs of a paper mill; suspected computer-generated content; unreliable results or conclusions; concerns about the data.

**Table 2:** Comparison of postoperative recovery-related indexes in each group ($\bar{x}$ ± *s*).

Indexes	Mild group (*n* = 54)	Moderate group (*n* = 42)	Severe group (*n* = 18)	*F*	*P*
Recovery time (min)	6.23 ± 2.15	8.96 ± 1.85^a^	11.24 ± 2.37^ab^	45.800	<0.001
Preoperative JOA score	11.26 ± 1.25	10.66 ± 1.03^a^	9.88 ± 1.08^ab^	10.420	<0.001
Postoperative JOA score	15.26 ± 2.25	14.83 ± 1.68	13.96 ± 3.01	1.550	0.216
Improvement rate	69.99 ± 22.85	65.77 ± 23.46	57.30 ± 20.15	2.140	0.122

*Note*. ^a^*P*  <  0.05 compared with the mild group; ^b^*P*  <  0.05 compared with the moderate group.

**Table 3:** Correlation analysis between severity of patients' condition and postoperative neurological recovery.

Indexes		Torg–Pavlov ratio	Spinal cord linear high-signal changes	First onset age	Disease duration
Postoperative JOA score	*r*	0.145	−0.158	0.169	0.177
	*P*	0.125	0.096	0.073	0.089

JOA score improvement rate	*r*	0.202	−0.199	0.080	0.187
	*P*	0.058	0.063	0.397	0.053

Postoperative recovery time	*r*	−0.250	0.505	−0.285	−0.532
	*P*	0.007	0.001	0.002	0.001

**Table 4:** Analysis of factors influencing the recovery time of postoperative neurological function.

Indexes	*β*	SE	Wald	*P*	OR	95% CI
Torg–Pavlov ratio	−1.154	0.845	6.389	0.012	0.849	0.152–0.967
Linear high-signal changes in the spinal cord	2.745	0.998	7.451	0.008	4.568	1.254–8.964
First onset age	−0.846	0.285	2.495	0.012	0.745	0.254–0.986
Duration of disease	−0.675	0.152	1.965	0.008	0.649	0.215–0.981

**Table 5:** ROC curve for predicting the recovery time of neurological function in patients with CSM.

Factors	AUC	Sensitivity	Specificity	*P*	95% CI
Torg–Pavlov ratio	0.794	75.20	75.60	0.000	0.692∼0.897
Linear high-signal changes in the spinal cord	0.767	74.10	79.20	0.000	0.662∼0.873
First onset age	0.772	80.05	69.40	0.000	0.664∼0.880
Duration of disease	0.801	81.80	79.40	0.000	0.696∼0.905
Joint detection	0.876	85.60	87.70	0.000	0.795∼0.957

## Data Availability

All data, models, and code generated or used during the study are available within the article.
